# Atypical nuclear localization of CD133 plasma membrane glycoprotein in rhabdomyosarcoma cell lines

**DOI:** 10.3892/ijmm.2015.2210

**Published:** 2015-05-14

**Authors:** ALENA NUNUKOVA, JAKUB NERADIL, JAN SKODA, JOSEF JAROS, ALES HAMPL, JAROSLAV STERBA, RENATA VESELSKA

**Affiliations:** 1 Department of Experimental Biology, Faculty of Science, Masaryk University, 61137 Brno, Czech Republic; 2 Regional Centre for Applied Molecular Oncology, Masaryk Memorial Cancer Institute, Masaryk University, 61137 Brno, Czech Republic; 3 Department of Pediatric Oncology, University Hospital Brno, Masaryk University, 61137 Brno, Czech Republic; 4 Department of Histology and Embryology, Faculty of Medicine, Masaryk University, 61137 Brno, Czech Republic

**Keywords:** CD133, prominin-1, rhabdomyosarcoma, cell nuclei, immunodetection

## Abstract

CD133 (also known as prominin-1) is a cell surface glycoprotein that is widely used for the identification of stem cells. Furthermore, its glycosylated epitope, AC133, has recently been discussed as a marker of cancer stem cells in various human malignancies. During our recent experiments on rhabdomyosarcomas (RMS), we unexpectedly identified an atypical nuclear localization of CD133 in a relatively stable subset of cells in five RMS cell lines established in our laboratory. To the best of our knowledge, this atypical localization of CD133 has not yet been proven or analyzed in detail in cancer cells. In the present study, we verified the nuclear localization of CD133 in RMS cells using three independent anti-CD133 antibodies, including both rabbit polyclonal and mouse monoclonal antibodies. Indirect immunofluorescence and confocal microscopy followed by software cross-section analysis, transmission electron microscopy and cell fractionation with immunoblotting were also employed, and all the results undeniably confirmed the presence of CD133 in the nuclei of stable minor subpopulations of all five RMS cell lines. The proportion of cells showing an exclusive nuclear localization of CD133 ranged from 3.4 to 7.5%, with only minor differences observed among the individual anti-CD133 antibodies. Although the role of CD133 in the cell nucleus remains unclear, these results clearly indicate that this atypical nuclear localization of CD133 in a minor subpopulation of cancer cells is a common phenomenon in RMS cell lines.

## Introduction

CD133 (also known as prominin-1) is a glycoprotein that is typically localized to the plasma membrane. The molecule consists of five transmembrane domains, two large extracellular loops, an extracellular N-terminus and an intracellular C-terminus. Eight potential glycosylation sites have been identified within the extracellular domains, with four per loop. Human CD133 is encoded by the *PROM1* gene, which is located in chromosomal region 4p15.32. At least seven CD133 isoforms resulting from alternative splicing have been described in humans (1,2).

CD133 is widely used to identify stem cells, and its glycosylated epitope, AC133, has recently been discussed as a marker of cancer stem cells (CSCs) in various human malignancies (2–4). In our previous studies, we identified CD133-positive cells that presented typical membrane positivity in two of the most common types of pediatric sarcomas, osteosarcoma (5) and rhabdomyosarcoma (RMS) (6). The expression of CD133 in these two solid tumors, as well as the tumorigenicity of CD133-positive cells, has been confirmed by other research groups (7–10). Therefore, CD133 is currently accepted as one of the markers of a CSC phenotype in pediatric sarcomas, including RMS (11–13).

During our recent study aimed at the analysis of CSC markers in pediatric sarcomas, we noted a surprising result: a stable subset of cells in each of five RMS cell lines examined exhibited an exclusive nuclear localization of CD133 (these data are published in this article). To date, a similar localization of this antigen has been described only in one case report of breast cancer (14) and in a large study on lung cancer (15) using immunohistochemical methods, nevertheless, without any verification or systematic description. For this reason, in this study, we sought to analyze this interesting phenomenon in detail using three independent anti-CD133 commercial antibodies (Fig. 1).

## Materials and methods

### Cell culture

Five cell lines derived from pediatric patients with RMS were included in this study: NSTS-8, NSTS-9, NSTS-11, NSTS-22 and NSTS-28. The first three cell lines were described in our previous study (6), and the last two were derived using the same procedure to generate primary cultures (16). All cell lines were authenticated by the immunodetection of MyoD, and the subtype was distinguished using *FKHR* break detection by fluorescence *in situ* hybridization (FISH). Authentication using MyoD detection was performed in the same passages as the experiments; FISH analysis of the *FKHR* break was completed up to passage 10. The cell lines were maintained in Dulbecco’s modified Eagle’s medium (DMEM) supplemented with 20% fetal calf serum, 2 mM glutamine, 100 IU/ml penicillin and 100 *µ*g/ml streptomycin (all purchased from GE Healthcare Europe GmbH, Freiburg, Germany). The cells were maintained under standard conditions at 37°C in a humified atmosphere containing 5% CO_2_ and were subcultured once or twice per week. The Research Ethics Committee of the School of Science (Masaryk University, Brno, Czech Republic) approved the study protocol, and a written statement of informed consent was obtained from each participant or his/her legal guardian prior to participation in this study. A brief description of the cohort of patients included in this study is provided in Table I.

### Indirect immunofluorescence

The cells were cultivated on coverslips in Petri dishes for one day and then rinsed with phosphate-buffered saline (PBS) and fixed with 3% paraformaldehyde (Sigma-Aldrich, St. Louis, MO, USA) at room temperature for 20 min. After washing again with PBS, nonspecific binding was blocked with 3% bovine serum albumin (BSA; Sigma-Aldrich) in PBS for 10 min. The cells were then incubated with primary antibody at 37°C for 60 min, washed three times in PBS and then incubated with the corresponding secondary antibody at 37°C for 45 min. Rabbit polyclonal anti-CD133 (Cat. no. ab19898, dilution 1:70; Abcam, Cambridge, UK), mouse monoclonal anti-CD133 (clone 17A6.1, Cat. no. MAB4399, dilution 1:100; Millipore, Billerica, MA, USA), mouse monoclonal anti-AC133 (clone AC133, Cat. no. 130-090-422, dilution 1:4; Miltenyi Biotec, Bergisch Gladbach, Germany), and mouse monoclonal anti-α-tubulin antibody (clone: TU-01, Cat. no. 11-250, dilution 1:100; Exbio, Vestec, Czech Republic), which served as a control, were used as the primary antibodies. Anti-rabbit Alexa Fluor 488 (Cat. no. A11008, dilution 1:200) and anti-mouse Alexa Fluor 488 antibody (Cat. no. A11001, dilution 1:200) (both from Invitrogen, Paisley, UK) were used as the secondary antibodies. After a final wash with PBS, the cell nuclei were counterstained with 0.05% Hoechst 33342 (Life Technologies, Carlsbad, CA, USA) for 10 min, and the coverslips were mounted using Dako fluorescence mounting medium (Dako, Glostrup, Denmark). An Olympus BX-51 microscope was used for sample evaluation; micrographs were captured using an Olympus DP72 CCD camera and analyzed using the Cell P imaging system (Olympus, Tokyo, Japan). At least 200 cells were evaluated overall within discrete areas of each sample, and the samples were prepared from at least three independent passages of all examined cell lines. The mean percentages of cells showing exclusive nuclear CD133 localization were determined for entire samples of individual cell lines. For the detailed examination of CD133 nuclear localization, the same protocol for indirect immunofluorescence was employed, and the specimens were then examined using an Olympus FluoView-500 confocal imaging system combined with an inverted Olympus IX-81 microscope. The images were recorded using an Olympus DP70 CCD camera and analyzed using analySIS FIVE software (Soft Imaging System GmbH, Muenster, Germany) and an Olympus FluoView Confocal Laser Scanning Microscope System 4.3.

### Transmission electron microscopy (TEM)

To perform the immunodetection of CD133 in ultrathin sections, the cells grown on coverslips were rinsed with PBS and fixed in 3% paraformaldehyde (Sigma-Aldrich) and 0.1% glutaraldehyde (AppliChem GmbH, Darmstadt, Germany) in PBS at room temperature for 60 min. Following a PBS rinse and dehydration, the cells were embedded in LR White medium (Polysciences Inc., London, UK). The labeling of the ultrathin sections was performed on grids. CD133 was detected using mouse monoclonal anti-CD133 antibody (dilution 1:25; Millipore) and a gold particle-conjugated secondary antibody (anti-mouse IgG 20 nm gold, Cat. no. ab27242, dilution 1:40; Abcam). Ultrathin sections incubated without primary antibody or with the TU-01 primary monoclonal antibody against α-tubulin (dilution 1:200; Exbio) were used as controls. Following immunodetection, the specimens were contrasted with 2.5% uranyl acetate (PLIVA-Lachema, Brno, Czech Republic) for 10 min and with Reynolds solution (Sigma-Aldrich) for 6 min at room temperature. The specimens were then observed under a Morgagni 268(D) transmission electron microscope (FEI Co., Hillsboro, OR, USA). The images were captured using an Olympus Veleta TEM CCD camera and analyzed using iTEM Olympus Soft Imaging Solution (Olympus).

### Immunoblot analysis

To analyze the nuclear and cytoplasmic fractions, a Nuclear Protein Extraction kit (Thermo Fisher Scientific, Rockford, IL, USA) was used according to the manufacturer’s instructions. A 20 *µ*l sample of protein extract was loaded onto an 8% sodium dodecyl sulfate (SDS)-polyacrylamide gel and separated by electrophoresis. Subsequently, the proteins were transferred onto polyvinylidene difluoride (PVDF) membranes (Bio-Rad Laboratories, Hercules, CA, USA), blocked in 5% non-fat milk at room temperature for 60 min, and incubated with primary antibodies, rabbit polyclonal anti-CD133 (Abcam), mouse monoclonal anti-α-tubulin (Exbio), or rabbit monoclonal anti-lamin B2 antibody (clone: D8P3U, Cat. no. 12255S; Cell Signaling Technology, Danvers, MA, USA) at a 1:1,000 dilution overnight at 4°C. Anti-α-tubulin and anti-lamin B2 served as the controls for the purity of the cytoplasmic and nuclear cell fractions, respectively. After washing with Tris-buffered saline (TBS)-Tween-20, the membranes were incubated with the corresponding horseradish peroxidase (HRP)-conjugated secondary antibodies anti-mouse IgG-HRP (cat. no. A9917, dilution 1:5,000; Sigma-Aldrich) and anti-rabbit IgG-HRP antibodies (cat. no. 7074, dilution 1:5,000; Cell Signaling Technology) at room temperature for 60 min. Signal detection was performed using ECL Prime Western Blotting Detection Reagent (GE Healthcare) according to the manufacturer’s instructions.

## Results

For all five RMS cell lines examined in this study, we performed a detailed analysis of the presence of cells with nuclear CD133 positivity using indirect immunofluorescence with three independent anti-CD133 antibodies (Fig. 1). A subset of cells showed only nuclear CD133 positivity, i.e., no detectable membrane or cytoplasmic positive signal. The results were markedly similar in all five cell lines analyzed, regardless of the primary antibody utilized, and the proportion ranged from 3.4 to 7.5%, with only minor differences observed among the individual anti-CD133 antibodies (Fig. 2A and Table I). We also performed a detailed morphological analysis of the cells that exhibited exclusive nuclear positivity for CD133 (Fig. 2B); as can be seen on these micrographs, the pattern of CD133 nuclear positivity was markedly similar in all of the cell lines.

To confirm the presence of CD133 in the nuclei of the RMS cells visualized using indirect immunofluorescence, we employed confocal microscopy and software cross-section analysis through these CD133-positive nuclei (Fig. 3). As is apparent from the results, the localization of the fluorescence signal for CD133 was detected within the cell nuclei both on the software cross-sections (Fig. 3B) and on the plot diagrams of the fluorescence intensity (Fig. 3D).

Furthermore, we also used immunogold labeling with TEM to verify the localization of CD133 in the nuclei of the RMS cells. To avoid any artifacts associated with this methodological approach, the accumulation of three or more gold particles together was considered to indicate a positive signal. The results clearly indicated the presence of CD133 in both the nuclei and nucleoli (Fig. 4A and B).

These results are all completely consistent with the microscopic observations described above (Fig. 2): the software cross-sections also showed clear, punctuate signals for CD133 within the nucleus (Fig. 3B and D), i.e., no diffuse positivity throughout the entire nucleus was observed. Nevertheless, the TEM micrographs also showed the presence of CD133 in the nucleoli (Fig. 4B), and this observation corresponds with the diffuse positivity for CD133 observed in some of the nucleoli (Fig. 2B). In addition to cells with the typical membrane positivity or exclusive nuclear positivity for CD133, we also sporadically noted clusters of positive signals in the cytoplasm near the cell nucleus or very close to the nuclear envelope (Fig. 4B).

Final confirmation of the results achieved through microscopic methods was carried out by immunoblot analysis of the cytoplasmic and nuclear fractions of all five RMS cell lines. The presence of CD133-specific bands of various intensities was detected in all nuclear fractions, in addition to the strong CD133-specific bands in the cytoplasmic fractions (Fig. 4C). The purity of both subcellular fractions was confirmed by the presence/absence of α-tubulin and lamin B2. These results are completely in accordance with our other findings (reported above) achieved by indirect immunofluorescence and TEM, i.e., in all five RMS cell lines, the presence of a small subpopulation of cells with CD133 in the nucleus was revealed.

## Discussion

As described above, we unexpectedly identified an atypical nuclear localization of CD133 in a relatively stable subset of cells in five RMS cell lines established in our laboratory. To date, this atypical localization of CD133 was described in one case report on breast cancer (14) and in a large study of prognostic markers on lung cancer (15) using immunohistochemical methods. Nevertheless, published data on CD133 expression in human cancer cells are partly inconsistent, possibly due to different analytical tools, as well as methodological limitations and pitfalls (2). For this reason, results obtained by immunohistochemistry or flow cytometry must be confirmed with alternative antibodies and should be complemented by the utilization of different detection methods of either protein or transcript (2). Furthermore, the glycosylation of CD133 epitopes in relation to the CSC phenotype should be also taken into account, particularly if the antibodies against AC133 epitope are commercially available (17).

In this study, we verified the nuclear localization of CD133 in RMS cells using three independent anti-CD133 antibodies, including both rabbit polyclonal and mouse monoclonal antibodies (Fig. 1). Indirect immunofluorescence and confocal microscopy followed by software cross-section analysis, TEM and cell fractionation with immunoblotting were also employed, and all the results undeniably confirmed the presence of CD133 in the nuclei of stable minor subpopulations of all five RMS cell lines.

These results strongly support the hypothesis that a stable subpopulation of cells with nuclear positivity for CD133 is a common phenomenon in RMS cell lines. Surprisingly, and to the best of our knowledge, similar results have not been reported to date for RMS cells. Although certain micrographs from our previous study showed cells with an accumulation of fluorescent signal for CD133 in the nucleus (6), we assumed that this finding was an artifact resulting from the use of a rabbit polyclonal antibody against CD133, (which was the only anti-CD133 antibody available at the time), although we had never detected similar nuclear positivity for CD133 in osteosarcoma or glioblastoma cell lines using the same antibody (5,18). Other authors investigating CD133 expression in RMS and RMS cell lines have not described the pattern of CD133 positivity in detail, and no micrographs of the individual cells are available in their published articles (9,10).

Very recently, one publication has mentioned the nuclear localization of CD133 in triple-negative breast cancer cells as revealed by immunohistochemistry; nevertheless, this study is a case report based on only one simple descriptive method and therefore does not include any continuing systematic analysis of this apparently interesting finding. Moreover, two of three methods listed in this article, quantitative RT-PCR and flow cytometry, are not suitable for identifying the cell surface, cytoplasmic or nuclear localization of any protein (14).

To date, another study concerning the possible value of CD133 as a prognostic indicator of survival in patients with non-small cell lung cancer (NSCLC) was just published. These interesting results suggest that CD133 expression in the nucleus of NSCLC cells was related to tumor diameter, tumor differentiation and the TNM stage. Kaplan-Meier survival and Cox regression analyses revealed that a high CD133 expression in the nucleus, as well as in the cytoplasm also predicted the poor prognosis of NSCLC (15).

As mentioned above, in addition to cells with the typical membrane positivity or exclusive nuclear positivity for CD133, clusters of positive signals in the cytoplasm near the cell nucleus or very close to the nuclear envelope were also sporadically noted. This finding is in accordance with our previously published observations of sporadic cytoplasmic positivity for CD133 in RMS cells (6), as well as with the deposition of CD133 in cytoplasmic vesicles that has been described in osteosarcoma (19) and the recently suggested mechanism of CD133 internalization and trafficking into lysosomes through interactions between CD133 and the histone deacetylase HDAC6 (20).

Taken together, our results undeniably confirmed the presence of CD133 in the cell nuclei of stable minor subpopulations in RMS cell lines. These results, although surprising and novel, were achieved through three independent methods using three independent antibodies purchased from three separate suppliers.

Nevertheless, the main question of what is the exact role of CD133 in the nucleus of RMS cells remains unanswered. In a previous study on breast cancer, the authors suggested that CD133 in the nucleus may act as transcriptional regulator and is most likely associated with a poor prognosis; however, this conclusion is largely speculative in this case report (14). By contrast, the most recent findings on NSCLC undoubtedly proved the association of nuclear positivity for CD133 poor prognosis in these patients (15).

Although a similar function of another type of surface molecule internalized into the cell nucleus, receptor tyrosine kinases, has been reported (21–23), CD133 belongs to a distinct class of cell membrane proteins, and the analogies to this process are therefore limited. Furthermore, recent studies also discuss the involvement of internalized CD133 in cell signaling pathways, such as the canonical Wnt pathway (20), or report an association between CD133 and the PI3K/Akt pathway (24–26). Regardless, the elucidation of the possible role of CD133 in the nucleus of cancer cells should be based on detailed descriptions of the localization and interactions of CD133 with other molecules in the cell nucleus. These experiments will be the focus of our upcoming study on this interesting phenomenon.

## Figures and Tables

**Figure 1:** Overview of epitopes of the anti-CD133 and anti-AC133 antibodies used in this study. For each antibody, the catalogue number and manufacturer are indicated. Potential glycosylation sites, as well as length of the N-terminal region, the intracellular and extracellular loops and the C-terminal region of CD133 are depicted.

**Figure 2:** Nuclear localization of CD133 in rhabdomyosarcoma cells. (A) Example of the frequency of cells with CD133 nuclear positivity in the NSTS-11 cell line, as detected using three independent primary antibodies. Cells with exclusive nuclear positivity for CD133 are indicated by arrows; cells with the typical membrane positivity are indicated by arrowheads. (B) Details of cells that exhibited exclusive nuclear positivity for CD133 in all five rhabdomyosarcoma cell lines. CD133 was stained by indirect immunofluorescence using Alexa Fluor 488-labeled secondary antibodies (green), and the nuclei were counterstained with Hoechst 33342 (blue). Scale bars, (A) 50 *µ*m and (B) 10 *µ*m.

**Figure 3:** Confocal microscopy analysis of CD133-positive cell nuclei. (A) The planes of software cross-sections through the CD133-positive nuclei are highlighted by simple yellow lines. (B) The cross-sections at these yellow lines are shown at the bottom. (C) The yellow arrows indicate lines drawn across individual CD133-positive nuclei in the confocal image; (D) matching plots reporting the fluorescence intensity according to these arrows are given below. CD133 was stained by indirect immunofluorescence using Alexa Fluor 488-labeled secondary antibodies (green), and nuclei were counterstained with Hoechst 33342 (blue). Scale bars, 5 *µ*m.

**Figure 4:** Detection of CD133 in the nuclei of rhabdomyosarcoma cells using transmission electron microscopy and immunoblot analysis. (A) Presence of CD133 in cell nuclei and nucleoli; more detailed images of the positive signal for CD133 in the highlighted square areas are presented on the bottom row. (B) The presence of CD133 in the cytoplasm near the nucleus (dashed square) and very close to the nuclear envelope (solid square). More detailed images of the positive signal for CD133 in the highlighted square areas, as indicated above, are shown on the right side. Representative labeling of CD133 in NSTS-28 cells is shown; CD133 was detected using 20 nm gold particles. Scale bars: (A) 250 nm and (B) 500 nm. (C) Nuclear/cytoplasmic fractionation followed by immunoblotting was performed using a rabbit polyclonal anti-CD133 primary antibody; α-tubulin and lamin B2 were used to confirm the purity of the fractions.

**Table I:** Description of patients from whom tumor samples were obtained to establish the rhabdomyosarcoma cell lines and the results concerning the mean percentage of cells with an exclusive nuclear localization of CD133.

Cell line	Gender	Age (years)	RMS type	No. of passages analyzed	Mean percentage of cells with exclusive nuclear localization of CD133		
					Anti-CD133 antibody (rabbit polyclonal)	Anti-CD133 antibody (mouse monoclonal)	Anti-AC133 antibody (mouse monoclonal)
NSTS-8	F	21	A	15–18	4.6	6.1	3.4
NSTS-9	M	17	A	13–18	4.6	5.2	4.1
NSTS-11	F	16	E	11–19	3.8	4.6	6.6
NSTS-22	F	5	A	11–15	4.0	6.0	6.4
NSTS-28	M	8	A	12–16	4.1	5.2	7.5

M, male; F, female; RMS, rhabdomyosarcoma. Tumor type: A, alveolar; E, embryonal.

## Abbreviations

BSA: bovine serum albumin
CSCs: cancer stem cells
DMEM: Dulbecco’s modified Eagle’s medium
FISH: fluorescence *in situ* hybridization
HRP: horseradish peroxidase
NSCLC: non-small cell lung cancer
PBS: phosphate-buffered saline
PVDF: polyvinylidene difluoride
RMS: rhabdomyosarcoma
SDS: sodium dodecyl sulfate
TBS: Tris-buffered saline
TEM: transmission electron microscopy
